The article "Transcriptional Repressor Gfi1 Integrates Cytokine-Receptor Signals Controlling B-Cell Differentiation" was retracted in 2012. Reasons: unreliable images; concerns about the images.

# Transcriptional Repressor Gfi1 Integrates Cytokine-Receptor Signals Controlling B-Cell Differentiation

**DOI:** 10.1371/journal.pone.0000306

**Published:** 2007-03-21

**Authors:** Chozhavendan Rathinam, Christoph Klein

**Affiliations:** Department of Pediatric Hematology/Oncology, Hannover Medical School, Hannover, Germany; Rockefeller University, United States of America

## Abstract

Hematopoietic stem cell differentiation is specified by cytokines and transcription factors, but the mechanisms controlling instructive and permissive signalling networks are poorly understood. We provide evidence that CLP1-dependent IL7-receptor mediated B cell differentiation is critically controlled by the transcriptional repressor Gfi1. Gfi1-deficient progenitor B cells show global defects in IL7Rα-dependent signal cascades. Consequently, IL7-dependent trophic, proliferative and differentiation-inducing responses of progenitor B cells are perturbed. Gfi1 directly regulates expression levels of IL7Rα and indirectly controls STAT5 signalling via expression of SOCS3. Thus, Gfi1 selectively specifies IL7-dependent development of B cells from CLP1 progenitors, providing clues to the transcriptional networks integrating cytokine signals and lymphoid differentiation.

## Introduction

The specification of hematopoietic stem cell fate depends on the coordinated actions of cytokines and transcription factors, yet the integrative signals orchestrating transcriptional networks remain poorly understood. Distinct developmental stages of hematopoietic stem cell (HSC) differentiation pathways have been defined. HSC differentiate into common lymphoid (CLP) and common myeloid progenitor (CMP) cells that constitute early branching points of lymphoid and myeloid lineage commitment, respectively [1]. Recently, a second common lymphoid progenitor cell population (CLP2) with restricted lymphoid differentiation capacity has been characterized in TCR-α transgenic mice and proposed to represent early thymic immigrants [2]. There is evidence that early thymic progenitor cells in the thymus may derive in a CLP1- and IL7- independent pathway [3], [6]. Bone marrow B cell development originating from CLP follows a highly regulated process characterized by well defined maturation stages [4]. Bone marrow B cells in the adult mouse are supposed to originate from CLP1 cells in an IL7R-dependent pathway. IL7 mediates survival, expansion, and differentiation of progenitor B cells [5]–[10].

Gfi1 is a SNAG-domain-containing zinc-finger transcriptional repressor that was originally described to confer cytokine-independent growth in a T cell lymphoma line [11]. Gfi1 belongs to a family of proteins (named Gfi/Pag-3/Senseless) involved in cell fate determination and differentiation [12]. In the hematopoietic system, Gfi1 plays a key role in restricting HSC proliferation and preserving their functional integrity [13], [14], in controlling T cell differentiation [15], [16], and in determining the differentiation of neutrophils [17], [18] as well as dendritic cells [19]. We hypothesized that Gfi1 controls cytokine-dependent B cell differentiation. Here, we analyze the role of Gfi1 in B cell development and provide insights into the mechanisms governing the developmental dichotomy of early lymphoid progenitor cells and IL7-mediated signals.

The article "Transcriptional Repressor Gfi1 Integrates Cytokine-Receptor Signals Controlling B-Cell Differentiation" was retracted in 2012. Reasons: unreliable images; concerns about the images.

## Results

### Characterisation of early lymphoid development in Gfi1^−/−^ mice

To address the role of Gfi1 in early B cell development, we first analyzed the numbers of lymphoid progenitor cells in Gfi1^−/−^ and Gfi1^+/+^ mice. As previously reported [14], the number of CLP1 cells (Lin^−^Sca1^+^IL7Rα^+^ckit^low^) was drastically reduced in Gfi1^−/−^ mice (Fig. 1A upper and lower panels). In contrast, both presumptive CLP2 (Lin^−^Sca1^+^IL7Rα^+^ckit^−^B220^+^, Fig. 1A middle and lower panels) and ETP (Early Thymic Progenitors, Lin^−^CD44^+^CD25^−^CD4^low/−^ckit^+^) (Fig. 1B) were normal in relative and absolute numbers, suggesting that Gfi1 plays a role in the differentiation of CLP1 but not of CLP2 or ETP. To further assess a potential role of Gfi1 in early lymphoid development, we made use of a transgenic Gfi1^GFP/Gfi1^ reporter mouse that allows monitoring of the transcriptional activity of the Gfi1 locus. As shown in Fig. 1C, Gfi1 is expressed in HSC and CLP1, but not in presumptive CLP2 or ETP, indicating that the latter populations may develop in a Gfi1-independent pathway. Transcriptional activity of the Gfi1 locus was observed in bone marrow B cells at all stages of differentiation, particularly in progenitor B cells at Hardy fractions C–E (Fig. 1A). Furthermore, a dynamic expression pattern of Gfi1 was seen in vitro, when HSC were differentiated into B cells in the presence of IL7 and SCF (Fig. S1B).

**Figure 1:** Developmental dichotomy of CLP1 and presumptive CLP2 progenitor cells evidenced by analysis of Gfi1^−/−^ and Gfi1^GFP/+^ mice. A) FACS plots indicating relative decrease of CLP1 (upper panels) and normal numbers of presumptive CLP2 (middle panels) in Gfi1^−/−^ bone marrow cells. Cells were pregated on Lin^−^IL7Rα^+^ cells (upper panels) and Lin^−^IL7Rα^+^Sca1^+^CD19^−^ cells (middle panels), respectively. Bar diagrams indicating absolute numbers of CLP1 and CLP2 cells of Gfi1^−/−^ and Gfi1^+/+^ mice (lower panel, n = 3 mice). Lineage markers included CD4, CD8, CD11c, CD11b and B220. Flow-cytometric analysis was performed on pooled BM cells from 5 mice. Shown is a representative experiment of 3. B) FACS plots indicating relative increase of ETP in Gfi1^−/−^ thymus. Lin^−^CD25^−^CD44^+^ cells (upper panels) were gated (G1) and analysed for expression of c-kit and IL7Rα (lower panels). Experiments were performed on pooled thymi (n = 5 mice). Bar diagrams indicating absolute numbers of ETP of Gfi1^−/−^ and Gfi1^+/+^ mice (lower panel, n = 3 mice). The total number of thymocytes was decreased by ∼6 fold in Gfi1^−/−^ mice. Shown is a representative experiment of 3. C) Transcriptional activity of Gfi1 locus in hematopoietic progenitor cells and thymic B cells. Pooled bone marrow cells or thymocytes (n = 5) were analyzed for GFP expression in the following populations: LSK (HSC), Lin^−^IL7Rα^+^Sca1^low^c-kit^low^ (CLP1), Lin^−^IL7Rα^+^Sca1^+^c-kit^−^B220^+^CD19^−^ (CLP2) and Lin^−^CD25^−^IL7Rα^−^CD44^+^c-kit^+^ (ETP). Shaded histograms represent GFP fluorescence in Gfi1^+/GFP^ cells, open histograms represent autofluorescence of Gfi1^+/+^ cells. The GMFI (Geo Mean Fluorescence Intensity) of Gfi1^+/+^ (above) and Gfi1^+/GFP^ (below) cells is indicated. Data are representative of 3 independent experiments.

The article "Transcriptional Repressor Gfi1 Integrates Cytokine-Receptor Signals Controlling B-Cell Differentiation" was retracted in 2012. Reasons: unreliable images; concerns about the images.

As previously shown [17], total numbers of B220^+^ cells in the bone marrow of Gfi1^−/−^ mice were significantly reduced, when compared to wildtype control mice (Fig. 2A). Furthermore, Hardy fraction B, proposed to represent an IL7-sensitive stage in B cell development [20], appeared proportionally reduced (Fig. 2B, Table S1). Despite distinct differences (e.g. with respect to Hardy fractions D, E, F) the bone marrow B cell compartment of Gfi1^−/−^ mice is reminiscent of IL7^−/−^ mice showing an incomplete block in maturation [6], [9], [10], [21].

**Figure 2:** Analysis of bone marrow B cell development in Gfi1^−/−^ mice. A) Absolute numbers of B220^+^ bone marrow B lineage cells determined from bone marrow of both hind limbs (n = 4 mice). B) FACS plots indicating relative decrease of bone marrow progenitor B cells in Gfi1^−/−^ mice according to the Hardy classification. B220^+^CD43^+^ cells were gated (G1) and further analyzed for expression of CD24 and BP-1 (middle panel). B220^+^CD43^−^ cells were gated (G2) and analysed for expression of B220 and IgM (bottom panel). Flow cytometry was done in pooled cell suspensions (n = 5 mice). Shown is a representative experiment of 5.

### Defective in vitro differentiation of B cells

Gfi1^−/−^ mice are prone to inflammatory reactions characterized by increased systemic cytokine levels [17], [18] that might constitute extrinsic factors influencing B cell differentiation. In a subsequent series of experiments we therefore directly analyzed IL7-dependent early B cell development in vitro. We isolated Lin^−^Sca1^+^c-kit^+^ (LSK) cells from Gfi1^+/+^ and Gfi1^−/−^ mice and determined their potential to differentiate into B cells in the presence of the cytokines SCF and IL7. In this in-vitro differentiation system, based upon an initial expansion step using a stem cell cytokine cocktail (IL3, IL6, SCF, Flt3L and TPO), complete maturation of B220^+^IgM^+^ can be seen using Gfi1^+/+^ HSC. In contrast to Gfi1^+/+^ progenitor cells, few Gfi1^−/−^ LSK cells differentiated into B220^+^CD19^+^ (5% versus 32%) and B220^+^IgM^+^ (0.9% versus 21%) cells, respectively (Fig. 3A), suggesting that cytokine-induced B cell differentiation is impaired in the absence of Gfi1. To prove a cell autonomous and specific role for Gfi1, we transduced Gfi1^−/−^ LSK cells with retroviruses encoding Gfi1-GFP and GFP, respectively, and cultured these genetically modified cells in SCF and IL7 containing medium. As shown in Fig. 3B, only Gfi1-transduced progenitor cells, but not GFP-transduced control cells, differentiated into B220^+^IgM^+^ B cells. In complementary experiments, we also determined whether a specific downregulation of Gfi1 in wildtype B cells would affect in vitro B cell differentiation. LSK cells were transduced with lentiviral vectors encoding a specific shRNA directed against Gfi1 or “empty” vectors, respectively. As expected, a knockdown of Gfi1 significantly impaired in vitro B cell differentiation (Fig 3C & Fig. S2). Taken together, these experiments suggest that Gfi1 is a specific, intrinsic, and cell-autonomous factor necessary for B cell development in-vitro.

The article "Transcriptional Repressor Gfi1 Integrates Cytokine-Receptor Signals Controlling B-Cell Differentiation" was retracted in 2012. Reasons: unreliable images; concerns about the images.

**Figure 3:** Defective in-vitro differentiation of Gfi1^−/−^ B cells. A) FACS plot showing block in in vitro B cell development in the absence of Gfi1. HSC were differentiated using IL7 and SCF and analyzed for expression of B220 and CD19 (top panel) and for expression of B220 and IgM (bottom panel). Data are representative of 3 independent experiments. B) FACS plot indicating rescue of B cell differentiation upon retroviral gene transfer. LSK cells from Gfi1^−/−^ mice were isolated and transduced with retroviral constructs encoding GFP or Gfi1-GFP. Transduced cells were cultured in the presence of SCF and IL7 for 14 days and GFP-positive cells were analyzed for expression of B220 and IgM. Data are representative of 2 independent experiments. C) FACS plot showing decreased in vitro B cell development upon knockdown of Gfi1 in HSC. HSC were transduced with lentiviral constructs encoding Gfi1 specific shRNA. Transduced cells were cultured in the presence of SCF and IL7 for 14 days and analyzed for expression of CD19 and IgM. Cells transduced with lentiviral backbone served as controls. Data are representative of 2 independent experiments.

The article "Transcriptional Repressor Gfi1 Integrates Cytokine-Receptor Signals Controlling B-Cell Differentiation" was retracted in 2012. Reasons: unreliable images; concerns about the images.

### IL7-mediated signals in Gfi1^−/−^ progenitor B cells

To further assess the functional relevance of Gfi1 in orchestrating IL7Rα-dependent signal cascades, we next analyzed trophic and proliferative effects of IL7 signalling. LSK HSCs were incubated in the presence of various cytokine combinations acting on hematopoietic progenitor cells and their viability was measured by propidium iodide exclusion 48 hours later. In these experiments, we tested both LSK progenitor cells and CD48^−^CD150^+^ hematopoietic stem cells (HSCs) (45). Both progenitor cell populations expressed IL7Rα upon 48 hours of cytokine stimulation, while no IL7Rα expression could be detected at hour 0 (Fig. S3). Whereas a cytokine cocktail consisting of IL3, SCF, Flt3L, and IL6 maintained the viability of Gfi1^−/−^ progenitor cells, Gfi1^−/−^ cells cultured in the presence of IL7 died (Fig. 4A and Fig. S4), indicating that Gfi1 plays a specific role in IL7-mediated trophic effects. This was confirmed by RT-PCR analysis documenting deficient IL7-mediated upregulation of the mRNA encoding the antiapoptotic protein Bcl2 (Fig. 4B). To assess proliferative responses of Gfi1^−/−^ hematopoietic stem cells, LSK cells were labelled with CFSE and cultured in the presence of IL7 or SCF & IL7. As shown in Fig. 4C, both Gfi1^−/−^ and Gfi1^+/+^ HSC divided in the presence of SCF & IL7, documented by a decrease in fluorescence intensity. In contrast, IL7 did not induce proliferation in Gfi1^−/−^ HSC. Similar results were seen when CD48^−^CD150^+^ cells were analyzed (Fig. S5). In addition to antiapoptotic and proliferative effects, IL7 also induces a differentiation program in progenitor B cells. To quantify B cell differentiation in Gfi1^−/−^ and Gfi1^+/+^ cells on a clonal level, HSC were cultured on semisolid medium in the presence of various cytokine combinations. 14 days later, Colony-Forming-Units (CFU) were counted. Compared to Gfi1^+/+^ HSC, Gfi1^−/−^ HSC gave rise to slightly increased numbers of CFU (8750 versus 6650) when incubated in the presence of IL3, SCF, Flt3L, IL6, potentially reflecting increased cell cycle progression in Gfi1^−/−^ HSC (13). In contrast, IL7-induced growth of colonies was severely impaired in Gfi1^−/−^ HSC (175 versus 2200) (Fig. 4D & Fig. S6), suggesting that IL7Rα-mediated signals are globally ineffective in the absence of Gfi1.

The generation of the earliest B cell progenitors critically depends on the transcription factors E2A and EBF. Both factors co-ordinately orchestrate the expression of B cell specific genes and immunoglobulin heavy-chain gene rearrangement [22]–[24]. Pax5 is the decisive B lineage commitment factor that restricts the developmental options of early progenitors to the B cell pathway [25]. As an example of instructive effects of cytokines on transcription factors, IL7 directs commitment of CLP by upregulating expression of EBF [6], [7]. We reasoned that in the absence of Gfi1 the coordinated expression of key transcription factors might be disturbed and measured their expression levels in defined progenitor B cell populations by RT-PCR. E2A and EBF were transiently upregulated at the transition from Hardy fraction B to D in wildtype B progenitor cells, but not in Gfi1^−/−^ progenitor cells (Fig. 4E upper and middle panels). These data were confirmed in independent experiments using B cell progenitor cells defined by the expression of B220, CD19, and IgM (Fig. S7B). As a consequence of E2A and EBF expression in progenitor B cells, Pax-5 is upregulated at the transition from Hardy fraction C to D. In line with decreased upregulation of E2A and EBF, Pax-5 transcription was not induced in Gfi1^−/−^ B cell progenitors (Fig. 4E lower panel and Fig S7B). The number of CD19 positive B-lineage cells was also reduced in Gfi1^−/−^ mice (Fig. 4F), either as a consequence of decreased Pax5 expression, or due to defects in fraction B cells. Thus, in the hierarchy of the signal cascade, Gfi1 appears to function upstream of IL7-mediated transcriptional activity of E2A, EBF and Pax5. Taken together, we document that the response to IL7 is severely reduced in Gfi1^−/−^ B progenitor cells resulting in defective B cell differentiation.

The article "Transcriptional Repressor Gfi1 Integrates Cytokine-Receptor Signals Controlling B-Cell Differentiation" was retracted in 2012. Reasons: unreliable images; concerns about the images.

### STAT-signalling and negative circuits

In view of global IL7-unresponsiveness of Gfi1^−/−^ cells affecting trophic, proliferative, and differentiation-inducing cellular responses, we reasoned that Gfi1-deficiency affected early IL7Rα signalling events such as activation of the JAK/STAT pathway. We isolated B220^+^lin^−^ cells from Gfi1^−/−^ and Gfi1^+/+^ mice and determined the levels of STAT5 phosphorylation at various time points after IL7 stimulation by Western blot. Whereas total STAT5 protein was comparable between Gfi1^−/−^ and Gfi1^+/+ ^control cells, IL7-induced STAT5 phosphorylation was completely absent in Gfi1^−/−^ cells (Fig. 5A). Since Gfi1 represents a zinc finger molecule mediating transcriptional repression in the nucleus, direct effects on IL7Rα activation appeared unlikely. We therefore hypothesized that the balance of activating and inhibitory effects on JAK-STAT-signalling might be affected in the absence of Gfi1. We quantified expression levels of SOCS3, an inhibitor of STAT5 carrying a putative Gfi1/Gfi1B-binding site in its promoter [26]. Interestingly, baseline levels and IL7-induced expression levels of SOCS3 mRNA (Fig. 5B) and protein (Fig. 5C) appeared increased in Gfi1^−/−^ progenitor B cells when compared to Gfi1^+/+^ cells. This finding indicates that decreased IL7-mediated signalling may at least partially be caused by preponderance of negative feedback circuits. To directly assess the role of unleashed SOCS3 expression in early B cell development, we transduced HSC from wildtype mice with retroviral constructs encoding SOCS3, expanded sorted cells in the presence of IL3, IL6, SCF, and Flt3L and evaluated IL7R-dependent signals. As shown in Fig 5D, transduced cells showed evidence of increased SOCS3 levels (upper panel). When SOCS3-overexpressing cells were stimulated by IL7, SOCS3-transduced progenitor cells revealed decreased phosphorylation of STAT5, as shown by intracytoplasmic FACS analysis (lower panel). In line with this observation, SOCS3-transduced cells also lost viability in response to IL7, whereas most control-transduced cells maintained their viability (Fig. 5E). These experiments show that elevated levels of SOCS3 are associated with decreased cellular responses to IL7 and thus provide mechanistic insights into the role of Gfi1 in negative feedback circuits controlling B cell differentiation.

The article "Transcriptional Repressor Gfi1 Integrates Cytokine-Receptor Signals Controlling B-Cell Differentiation" was retracted in 2012. Reasons: unreliable images; concerns about the images.

**Figure 4:** Defective IL7Rα signalling in Gfi1^−/−^ progenitor cells. A) Viability of HSC in response to hematopoietic growth factors. LSK cells from Gfi1^+/+^ and Gfi1^−/−^ mice were initially cultured in the presence of SCF, IL6, IL3, TPO and Flt3L for 48 hours and subsequently cultured in the presence of indicated cytokines. Cells were analyzed by PI staining and FACS 48 hours later. Shown are the mean values of duplicate samples. Data are representative of 2 independent experiments. B) Realtime PCR showing Bcl2 RNA levels. Sorted Lin−B220+ bone marrow cells were stimulated with IL7. RNA was extracted at indicated time points and reverse transcribed into cDNA. Shown are the mean values of duplicate samples. Data are representative of 2 independent experiments. C) Cell proliferation indicated by CSFE dilution. LSK cells from Gfi1^+/+^ and Gfi1^−/−^ mice were initially cultured in the presence of SCF, IL6, IL3, TPO and Flt3L for 48 hours. Cells were washed, labeled with CSFE and incubated in the presence of indicated cytokines for 72 hours. Histograms representing CFSE fluorescence and division history of Gfi1^+/+^ (top panel) and Gfi1^−/−^ (bottom panel) cells are shown. Data are representative of 2 independent experiments. D) CFU assay indicating decreased colony-forming-activity in Gfi1^−/−^ HSC. LSK cells were cultured on semisolid medium in the presence of indicated cytokines. 14 days later, the absolute numbers of colony forming units of Gfi1^+/+^ (white bars) and Gfi1^−/−^ (black bars) cells were enumerated and plotted. Data are representative of 2 independent experiments. E) Expression of B cell specific transcription factors in defined precursor B cell populations according to Hardy classification. mRNA expression levels of E2A (top panel) EBF (middle panel) Pax5 (bottom panel) were determined by RT-PCR. Shown are the mean values of duplicate samples. Data are representative of 2 independent experiments. F) Contour plots indicating reduced expression of CD19 in Gfi1^−/−^ bone marrow B lineage cells (upper panels). Bar diagrams indicating absolute numbers of CD19^+^ cells in BM of Gfi1^−/−^ and Gfi1^+/+^ mice (lower panel, n = 3 mice). Data are representative of 6 independent experiments.

The article "Transcriptional Repressor Gfi1 Integrates Cytokine-Receptor Signals Controlling B-Cell Differentiation" was retracted in 2012. Reasons: unreliable images; concerns about the images.

**Figure 5:** Defective STAT5 signalling in Gfi1^−/−^ progenitor B cells. A) Western blot analysis showing decreased STAT5 phosphorylation in B220^+^ bone marrow cells upon IL7-signalling. Data are representative of 2 independent experiments. B) Realtime PCR showing increased RNA levels of SOCS3 in Gfi1^−/−^ B cells. Sorted B220^+^ bone marrow cells were stimulated with IL7, RNA was extracted at indicated time points and reverse transcribed into cDNA. Expression of SOCS3 mRNA was quantified by realtime PCR. Shown are the mean values of duplicate samples. Data are representative of 2 independent experiments. C) Western blot showing protein levels of SOCS3. Sorted B220^+^ bone marrow cells were stimulated with IL7 and assessed for SOCS3 protein using specific polyclonal antibodies. GAPDH was detected by specific monoclonal antibodies to confirm equal protein loading. Data are representative of 2 independent experiments. D) Intra-cytoplasmic detection of SOCS3 and p-STAT5 by FACS. LSK cells from Gfi1^+/+^ mice were transduced with either GFP or SOCS3-GFP retroviruses, respectively. SOCS3 expression was measured by cytoplasmic staining with an anti-SOCS3 monoclonal antibody (upper panel). Sorted GFP and SOCS3-GFP transduced progenitor cells were stimulated in the presence of IL7 for 10 minutes and intra cytoplasmic staining was performed using an anti-pSTAT5 monoclonal antibody (lower panel). Shaded histograms represent cells stained with isotype control antibodies. Data are representative of 2 independent experiments. E) Viability of SOCS3 over-expressing progenitor cells in response to IL7. Sorted GFP and SOCS3-GFP transduced progenitor cells were cultured in vitro in the presence of IL7. At indicated timepoints, cells were analyzed by PI staining and FACS. Shown are the mean values of duplicate samples. Data are representative of 2 independent experiments.

The article "Transcriptional Repressor Gfi1 Integrates Cytokine-Receptor Signals Controlling B-Cell Differentiation" was retracted in 2012. Reasons: unreliable images; concerns about the images.

### Modulation of IL7Rα-expression

Coordinated lymphocyte development is not only critically dependent on IL7-mediated signals but also on dynamic and developmental-stage-specific regulation of the IL7Rα chain [27]–[31]. Since the IL7Rα gene contains putative binding sites for Gfi1 [32], we analyzed IL7Rα expression levels in distinct progenitor B cells in vivo. As shown in Fig. 6A, Gfi1^−/−^ progenitor B cells at Hardy fractions D and E showed a higher mean fluorescence index of IL7Rα compared to Gfi1^+/+^ control cells. This finding was confirmed in independent experiments using CD19 as an unambiguous marker of the B cell lineage (Fig. S8). Similar differences were seen in an in-vitro differentiation system allowing the simultaneous detection of IL7Rα mRNA and cell surface expression (Fig. 6 B,C). These results suggest that Gfi1 directly represses IL7Rα transcription and thus allows coordinated B cell development to proceed. To directly prove binding of Gfi1 to a cognate binding site in the IL7Rα gene, we performed chromatin-immunoprecipitation studies in progenitor B cell extracts from Gfi1^+/+^ mice. As shown in Fig. 6 D and E, direct binding of Gfi1 could be documented to a Gfi1-binding site in intron 2 of IL7Rα, but not to putative Gfi1 binding sites present in intron 3, intron 4, or the promoter. This indicates that the IL7Rα gene is a direct target of the transcriptional repressor Gfi1. Thus, we define a complex mechanistic role for Gfi1 in IL7-mediated signalling as well as in direct downregulation of IL7Rα.

**Figure 6:** Modulation of IL7Rα expression by Gfi-1. A) Histograms plots indicating IL7Rα surface expression in distinct populations of bone marrow B lineage precursor cells. BM cells from 5 mice were pooled, and IL7Rα expression was analyzed in the following subpopulations: B220^+^CD43^+^BP1^−^CD24^−^ (Fraction A), B220^+^CD43^+^CD24^+^ (Fraction B–C), B220^+^CD43^−^IgM^−^ (Fraction D), B220^+^CD43^−^IgM^+^ (Fraction E), and B220^high^CD43^−^IgM^high^ (Fraction F). Shaded histograms represent IL7Rα fluorescence and open histograms represent isotype fluorescence. The GMFI_i_ is indicated in each plot. Geometric mean fluorescence intensity index was calculated as follows: GMFI_i_ = GMFI_(antibody stained cells)_−GMFI_(Isotype control treated cells)_. Data are representative of 5 independent experiments. B–C) Realtime PCR showing IL7Rα RNA and surface expression levels during in vitro B cell development. LSK bone marrow cells isolated from Gfi1^+/+^ and Gfi1^−/−^ mice were first expanded for 48 hours in a cytokine cocktail containing IL3, IL6, SCF, Flt3L, TPO and then cultured in the presence of SCF and IL7. RNA was extracted at indicated time points, reverse transcribed into cDNA and Realtime PCR was performed (B). Cell surface expression of IL7Rα during in vitro B cell differentiation. LSK bone marrow cells of Gfi1^+/+^ and Gfi1^−/−^ mice were cultured in the presence of SCF and IL7. Aliquots of cells were taken at indicated time points and analyzed for expression of IL7Rα by FACS (C). Shown are the mean values of duplicate samples. Data are representative of 2 independent experiments. D) Chromatin-immunoprecipitation analysis of Gfi1 binding to the IL7Rα gene. Crosslinked chromatin from Gfi1^+/+^ bone marrow B220^+^ cells was immunoprecipitated using control goat IgG or anti-Gfi1 antibodies. PCR was performed on input DNA and immunoprecipitated DNA using primer pairs spanning Gfi1 binding sites that are present in intron 2, intron 3, intron 4, promoter and exon 8 of the IL7Rα gene, respectively. Genomic DNA and no template lanes represent controls. Data are representative of 2 independent experiments. E) Semi-quantitative real time PCR analysis. Crosslinked chromatin from Gfi1^+/+^ and Gfi1^−/−^ bone marrow B220^+^ cells was immunoprecipitated using control goat IgG or anti-Gfi1 antibodies. Realtime PCR was performed on input and immunoprecipitated DNA using primer pairs spanning Gfi1 binding sites in intron 2 of IL7Rα gene. Data are representative of 2 independent experiments.

The article "Transcriptional Repressor Gfi1 Integrates Cytokine-Receptor Signals Controlling B-Cell Differentiation" was retracted in 2012. Reasons: unreliable images; concerns about the images.

## Discussion

We have shown that Gfi1 is a critical modulator of IL7-dependent B cell differentiation. Gfi1 is selectively expressed in CLP1 cells but not in presumptive CLP2 cells and controls IL7-dependent signals in B progenitor cells in bone marrow. IL7-mediated signals require integration via Gfi1 since transcriptional repression of inhibitory circuit factors and IL7Rα are critically dependent on Gfi1. Thus, the analysis of Gfi1^−/−^ mice has shed light on a number of important questions regarding controversial issues in early lymphoid and B cell development.

The identification of CLP2 cells in pre-TCR-α transgenic reporter mice [2] has led to a recent refinement in the understanding of early lymphoid development. Since the nature of CLP2 cells remains controversial, we have defined Lin^−^Sca1^+^IL7Ra^+^ckit^−^B220^+^ cells as “presumptive” CLP2 cells and attempted to elucidate transcriptional networks controlling the specification of CLP1 versus CLP2 cells. A detailed analysis of Ikaros^−/−^ mice that show evidence of ongoing thymopoiesis without bone marrow B cell development revealed normal frequencies of ETPs and absence of classical bone marrow CLPs [3]. Even though this phenotype shares certain similarities to Gfi1^−/−^ mice, it is not known whether Ikaros specifies CLP1 versus CLP2. In this respect, the observation that Gfi1 is differentially expressed in CLP1 versus presumptive CLP2 cells is interesting in light of the recently documented existence of independent B cell lineages [33], [34].

The article "Transcriptional Repressor Gfi1 Integrates Cytokine-Receptor Signals Controlling B-Cell Differentiation" was retracted in 2012. Reasons: unreliable images; concerns about the images.

IL7 is a critical factor for survival, expansion, and differentiation of progenitor B cells in adult mice [5]–[10]. Both IL7^−/−^ and IL7Rα^−/−^ mice demonstrate lymphopenia associated with an incomplete block in B cell development [9], [10]. In IL7^−/−^ mice, bone marrow production of B cells ceases after 8 weeks of age, while a pool of mature B cells is sustained that has been proposed to derive from IL7-independent fetal or perinatal precursor B cells [21]–[35].

Our analysis of Gfi1^−/−^ B cell compartments revealed certain similarities between Gfi1^−/−^ and IL7^−/−^ progenitor B cells, suggesting that both IL7 and Gfi1 may act via a common pathway. However, Gfi1^−/−^ mice and IL7^−/−^ are not identical with respect to their B cell phenotype. For example, CLP1 cells are present in IL7^−/−^ mice [7] and severely reduced in Gfi1^−/−^ mice. We found that multiple IL7-mediated effects in progenitor B cells are severely reduced in the absence of Gfi1. Perhaps most significantly, IL7-induced upregulation of E2A, EBF, and Pax5, critical transcription factors controlling B cell differentiation, is severely perturbed. It should be noted however, that these effects may not be completely dependent on defective IL7-mediated signals but may result from as yet undefined other roles of Gfi1. In this respect, IL7R^−/−^ mice show normal levels of E2A [7], suggesting that E2A is controlled by mechanisms other than IL7. Nevertheless, the net effect of decreased IL7Rα-dependent signals may at least partially account for a block in B cell development implying that Gfi1 is critically important in IL7-dependent B cell differentiation.

Our findings are also relevant for an ongoing controversy bearing on the dichotomy of B1 versus B2 cells. Whereas conventional B2 cell differentiation is affected in Gfi1-deficient mice, our data suggest that B1 cell differentiation might be preserved (Rathinam and Klein, submitted). Thus, similar to PU.1 [36], [37], Gfi1 may be involved in the specification of distinct developmental fates in B cell differentiation. Recently, a B1 B cell specific progenitor has been identified in fetal and adult bone marrow [33], further supporting the concept that B1 and B2 cell differentiation represent distinct lineages.

Gfi1 is a transcriptional repressor binding to cognate binding sequences in regulatory elements [38], [39]. The precise mechanism of action is under active investigation. Gfi1 and its homologue Gfi1B share a DNA binding and a SNAG (Snail and Gfi1 family of proteins) domain mediating transcriptional repression of multiple target genes, including Gfi1 itself [38], [40]. We have provided evidence for two independent and mutually non-exclusive mechanisms accounting for decreased B cell development in Gfi1^−/−^ mice, i.e. i) regulation of negative feedback loops and ii) deficient downregulation of IL7Rα. Indirect effects of Gfi1 on cytokine receptor signalling have been shown previously in myeloid development, where impaired STAT3 signalling in Gfi1^−/−^ precursor dendritic cells has been associated with increased transcription of PIAS3 and SOCS3 [19]. Here, we provide evidence that similar feedback mechanisms control early B cell development by integrating cytokine signals and negative circuit loops. Our data indicate that IL7-dependent STAT5 signalling is decreased in the absence of Gfi1. We cannot definitively exclude the concern that our data of decreased STAT5 phosphorylation and increased SOCS mRNA and protein levels may be confounded by the fact that the Gfi1^+/+^ and Gfi1^−/−^ cell populations differ in various respects. However, SOCS3 gene transfer experiments into wildtype cells recapitulate the scenario of decreased IL7-mediated survival signals, and dysbalanced expression levels of negative feedback regulators has also been observed in Gfi1^−/−^ myeloid cells [19].

The article "Transcriptional Repressor Gfi1 Integrates Cytokine-Receptor Signals Controlling B-Cell Differentiation" was retracted in 2012. Reasons: unreliable images; concerns about the images.

Furthermore, the coordinated development of lymphoid cells is dependent on tightly regulated expression levels of IL7Rα. High levels of IL7Rα lead to a block in B cell development whereas low levels are permissive for B cell development [31]. In addition, at the proB to preB transition, diminishing IL7-mediated signals may permit selective expansion of B cells [28]. However, the mechanisms regulating IL7Rα expression remain largely unknown. Gfi1^−/−^ progenitor B cells showed increased levels of IL7Rα expression in vivo and in vitro, suggesting that defects in quantitative calibration of IL7Rα signal transduction may at least partially contribute to perturbed B cell differentiation. In progenitor B cells, PU.1 has been shown to bind to IL7Rα promoter sequences, thus controlling early lymphoid development via IL7Rα expression [41]. In CD8 T cells, IL7Rα transcription is suppressed by IL7 in a Gfi1-dependent manner [32], suggesting that Gfi1 may also modulate IL7Rα expression. Furthermore, transgenic Gfi1B expression leads to defects in IL7Rα expression [15]. The murine IL7Rα a gene contains several putative Gfi1 consensus binding sites. We now could demonstrate directly by chromatin-immunoprecipitation experiments that Gfi1 binds to a cognate site in intron 2. Taken together, our findings suggest that Gfi1 directly represses IL7Rα expression in progenitor B cells. Since IL7Rα expression is a phenotypic hallmark of early lymphoid progenitor cells, this finding is of relevance with respect to the interpretation of the phenotypic characterisation of progenitor B cells in Gfi1-deficient mice. However, at the hematopoietic progenitor cell level, IL7Rα expression is not changed in Gfi1^−/−^ mice (Fig. 6A and Fig. S3), suggesting that additional factors may contribute to differences in IL7Rα levels in lymphoid progenitor cells.

The article "Transcriptional Repressor Gfi1 Integrates Cytokine-Receptor Signals Controlling B-Cell Differentiation" was retracted in 2012. Reasons: unreliable images; concerns about the images.

In summary, we provide evidence that Gfi1 provides an important link between cytokine signalling and transcriptional regulation by modulating cytokine-receptor signalling. These insights open a new perspective for understanding lymphoid development in health and disease, B-cell mediated pathology, and potential therapeutic manipulations of cytokine-controlled transcription factor networks.

## Materials and Methods

### Mice

All mice were bred and maintained under specific pathogen free conditions in the central animal facility at Hannover Medical School. Gfi1^−/−^ mice [18] and Gfi1^GFP/+^ mice [42] were kindly provided by Tarik Möröy, Essen. Both mouse strains were backcrossed on C57/BL6 background for >8 generations. In Gfi1^GFP/+^ reporter mice, exons 1–7 of Gfi1 have been replaced by the GFP cDNA, their phenotype is similar to wildtype mice. In all experiments, age and sex matched mice were used at four to eight weeks of age. All experiments were approved by the institutional review board.

### Cells and cell culture

In vitro cultures were performed using purified either LSK (Lin^−^Sca-1^+^c-kit^+^) or CD150^+^CD48^−^ cells that were described recently (45). For sorting of CD150^+^CD48^−^ cells, RBC depleted total BM cells were stained with 1 ug (per 1×10^6^ cells) of biotin conjugated anti CD48 and PE conjugated anti CD150 antibodies for 15 minutes on ice. For secondary staining, cells were washed twice with PBS 2% FCS and stained with 0.25ug (per 1×10^6^ cells) APC conjugated streptavidin antibodies, further incubated for 15 minutes and washed twice with PBS 2% FCS. Cells were resuspended in PBS 0.5% BSA and passed through nylon mesh prior to sorting. Cell sorting was performed with FACS Aria cell sorter and FACS Diva software. After every sorting, cells were reanalysed for checking its purity, and the purity was always >95%. and the following recombinant cytokines: 10 ng/ml rm-IL3, 10 ng/ml rm-IL6, 50 ng/ml rm-SCF, 50 ng/ml rh-Flt3L and 10 ng/ml rm-IL7 (all from Peprotech, Rocky Hill, NJ). To assess viability, cells were harvested after 48 hours, stained with 1 µg/mL of propidium iodide (Sigma Aldrich, Munich, Germany) and analysed by flow-cytometry. For in vitro proliferation experiments, LSK cells were sorted and labelled with 2 µM of CFDA-SE dye (Molecular probes, Karlsruhe, Germany) in 10 mL of PBS for 10 min at 37°C. Cells were washed and incubated in IMDM medium supplemented with 10% FCS, 2 mM L-Glutamine, 1% Penicillin-Streptomycin, 1 mM non-essential amino acids, 10 ng/ml rm-IL3, 10 ng/ml rm-IL6, 50 ng/ml rm-SCF, 50 ng/ml rh-Flt3L and 10 ng/ml rm-IL7 (all from Peprotech, Rocky Hill, NJ). After 72 hours of culture cells were harvested and analysed by flow-cytometry. For CFU assays, 1×10^5^ either LSK or CD150^+^CD48^−^ cells were mixed thoroughly with methocult (03234, CellSystems, St. Katharinen, Germany) and plated in the presence of the following cytokines: rm-IL3 (10 ng/ml), rm-IL6 (10 ng/ml), rm-SCF (50 ng/ml), rh-Flt3L (50 ng/ml) and rm-IL7 (10 ng/ml) (all from Peprotech, Rocky Hill, NJ). After 14 days of culture, colonies were counted using an inverted microscope (Axiovert-II Zeiss) and gridded scoring dishes.

The article "Transcriptional Repressor Gfi1 Integrates Cytokine-Receptor Signals Controlling B-Cell Differentiation" was retracted in 2012. Reasons: unreliable images; concerns about the images.

For in vivo B cell analysis, lymphoid organs were cut into small pieces, treated with collagenase D (Boehringer, Mannheim, Germany) for 30 min at 37°C, gently meshed and washed with PBS containing 50 µg/mL Dnase I (Roche, Mannheim, Germany) and 2 mM EDTA. In some experiments, BM B220^+^ cells were purified by labelling mononuclear cell suspensions with anti-CD45R microbeads (B220) and subsequent enrichment by immunomagnetic columns (Miltenyi Biotech, Bergisch Gladbach, Germany).

For retroviral gene transfer, Sca-1^+^lin^−^ cells were cultured in IMDM containing 10% FCS, 2 mM L-Glutamine, 1% Penicillin-Streptomycin, 1 mM Non-essential amino acids, 10 ng/ml rm-IL3, 10 ng/ml rm-IL6, 50 ng/ml rm-SCF, 50 ng/ml rh-Flt3L and 25 ng/ml h-TPO.

### BrdU assays

Purified HSCs were cultured as mentioned above. 60 uM of BrdU (Sigma) was added to cells and cultured for an additional 12 hours. Cells were washed and permeabilized with FACS permeabilizing solution (BDIS, San Jose, CA). Cells were stained with anti BrdU antibodies in the presence of DNase at RT for 60 minutes. Cells were washed and analyzed by flow cytometry.

### Flow cytometry

Single cell suspensions were analysed by flow cytometry using FACS SCAN or FACS Canto and CELLQuest software, FACS Diva software (BD Biosciences, San Jose, CA) or Flow Jo software (Tree Star, Inc., Ashland, OR), respectively. Cell sorting of defined subpopulations was performed using Moflo cell sorter (DAKO Cytomation, Glostrup, Denmark) or FACSAria cell sorter (BD Biosciences, San Jose, CA), respectively.

The following monoclonal antibodies (all from BD Pharmingen, San Diego, CA except noted otherwise) were used: CD3e-FITC, -biotin &-PEcyc7, CD4-FITC, -PE, -APC, CD8 -PerCP & -PE, CD11b-FITC & -biotin, CD19-PE, CD24-FITC, CD25-FITC & -PerCP, CD34-FITC, CD43-biotin, CD44-FITC & -PE, CD48-biotin, CD117-PE & -APC, CD150-PE, B220-FITC, -PE, -biotin & -APCcyc7, BP-1-PE, IgM-FITC, -APC & -PEcyc7, Gr-1-FITC & -biotin, IL-7Rα-biotin, Sca-1-PE, Flt3-PE, BrdU- FITC, TER119-biotin, anti-mouse-STAT5, anti-mouse-STAT5-p (Cell signalling technology, Frankfurt, Germany), anti-mouse-SOCS3 (Zymed Laboratories, South San Francisco, CA), Gfi1 (N20; Santa Cruz Biotechnology), goat-anti-mouse-IgG-HRP, goat-anti-rabbit-IgG-HRP (Cell signalling technology, Frankfurt, Germany). In all experiments, cells were also stained with corresponding isotype-matched monoclonal antibodies. Cells reacted with biotinylated monoclonal antibodies were incubated with fluorochrome-conjugated streptavidin-PerCP or streptavidin-APC (BD Pharmingen). All fluorescence intensity plots are shown in log scales.

The article "Transcriptional Repressor Gfi1 Integrates Cytokine-Receptor Signals Controlling B-Cell Differentiation" was retracted in 2012. Reasons: unreliable images; concerns about the images.

### Intracytoplasmic staining

To detect STAT5 phosphorylation and SOCS3 expression by flow cytometry, LSK cells transduced GFP or SOCS3 GFP were stimulated with rmIL-7 for 10 min. Cells were first fixed, permeabilized using a commercially available Fix and Perm kit (Caltag Laboratories, Burlingame, CA) and stained with anti-SOCS3 and p-STAT5 antibodies respectively. Cells were washed and stained with anti-mouse-IgG-FITC secondary antibodies and detected by flow cytometry.

### Protein assays

Extraction of proteins was carried out using standard protocols. Briefly, cells were harvested and lysed in hypotonic buffer containing 20 mM Hepes (pH 7.6), 10 mM KCl, 1 mM MgCl_2_, 2% glycerin, 0.1% Triton-X100, 0.5 mM DTT (Roche), 1 mM Pefabloc (Roche), 1 mM sodium-orthovandate (Sigma), 5 µg/mL protease inhibitor cocktail (Sigma). Nuclear and cytoplasmic protein fractions were separated by centrifugation (×1800g). The pellet containing nuclear proteins was re-suspended in hypertonic buffer containing 20 mM Hepes (pH 7.9), 400 mM NaCl, 1 mM EDTA, 20% Glycerin, 0.1% Triton-X, 0.5 mM DTT (Roche), 1 mM Pefabloc, 1 mM sodium-orthovandate, 5 µg/mL protease inhibitor cocktail and incubated for 15 min at 4°C. The lysate was subjected to centrifugation (×16,000g) and the supernatant containing the nuclear proteins was collected. Protein quantification was performed using Bradford reagent (Bio-rad, Munich, Germany). For Western blot analysis, 20 µg of protein was loaded on an 8% SDS gel, separated by electrophoresis and blotted onto nylon membranes. The membranes were exposed to anti-STAT-5, anti-STAT-5p and anti-SOCS3 respectively, followed by staining with secondary antibodies conjugated to horse radish peroxidase. The enzymatic reaction was visualized using ECL reagents (ECL kit, Amersham Biosciences, Freiburg, Germany).

The article "Transcriptional Repressor Gfi1 Integrates Cytokine-Receptor Signals Controlling B-Cell Differentiation" was retracted in 2012. Reasons: unreliable images; concerns about the images.

### RNA isolation and Real Time PCR

Total RNA was isolated using commercially available kit systems (“Absolutely RNA mini prep kit” - Stratagene, La Jolla, CA). cDNA was synthesised using oligo dT primer and expand reverse transcriptase (Roche). E2A, EBF and PAX5 expression was determined by Real Time PCR using the E2A specific forward primer 5′-TGACAGCTACAGCAGGGATG and reverse primer 5′-AGCGAGCCATTAACCTCAGA, EBF specific forward primer 5′ –CATGTCCTGGCAGTCTCTGA and reverse primer 5′-CAACTCACTCCAGACCAGCA, and Pax5 specific formard primer 5′- GAACTTGCCCATCAAGGTGT and reverse primer 5′-TGTCCGAATGATCCTGTTGA. SOCS3 expression was determined by Real Time PCR using a SOCS3 specific forward primer 5′-ATGGTCACCCACAGCAAGTT and reverse primer 5′-TGACGCTCAACGTGAAGAAG. Gfi1 mRNA expression in knock down studies was measured by RT-PCR using the specific forward primer 5′-CAGCTTACCGAGGCTCCCGACAGG and reverse primer 5′-CAAGACCGCTCCATGCATAGGGCTT. GAPDH specific primers were used as internal controls (forward primer 5′ GTCAGTGGTGGACCTGACC; reverse primer 5′-TGAGCTTGACAAAGTGGTCG). The PCR reaction was performed in duplicates using either a LightCycler–FastStart DNA Master SYBR Green I kit (Roche) or QuantiTect SYBR Green PCR Kit (Qiagen, Hilden, Germany) according to the manufacturer’s instructions.

### Retroviral gene transfer

The murine Gfi1 cDNA and SOCS3 cDNA were cloned into the retroviral vector SFβ-91-IRES-EGFP, kindly provided by C. Baum, Hannover. Recombinant VSV-G pseudotyped retroviruses were generated using transient transfection into the packaging cell line 293GPG (43). For retroviral gene transfer, LSK progenitor cells were stimulated for 48 hours in the presence of a stem cell cytokine cocktail (see above) and transduced at a multiplicity of infection (MOI) of 10 in the presence of 8 µg/ml polybrene (Sigma). In brief, cells were exposed to recombinant retrovirus for 1 hour at 37°C, followed by spinoculation for 2 hours at ×700 g and further incubation at 37°C in 5% C0_2_. Subsequently, cells were washed, cultured for additional 48 hours in the presence of the stem cell cytokine cocktail and used for in vitro experiments. The average transduction efficiency was 50–60%.

For shRNA studies, Gfi1 specific shRNAs were designed through VectorNTI (Invitrogen) software. Two shRNAs recognising Gfi1 specific mRNA at different regions (shRNA1 and shRNA2) were cloned into pSM2 (open biosystems) lentiviral backbone. Lentiviruses were generated using 293T cell lines and viral titer was determined by counting the puromycin resistant colonies. For knocking down Gfi1 mRNA, prestimulated LSK cells were transduced as mentioned above and transduced cells were cultured in the presence of SCF+ IL7 for 14 days either in the presence or absence of puromycin (1 µg/mL).

The article "Transcriptional Repressor Gfi1 Integrates Cytokine-Receptor Signals Controlling B-Cell Differentiation" was retracted in 2012. Reasons: unreliable images; concerns about the images.

### Chromatin-immunoprecipitation assay

Chromatin immunoprecipitation assays were performed as described (44) with few modifications. Cells (5–10×10^7^) were crosslinked for 10 min at room temperature by adding paraformaldehyde (1% final concentration). The crosslinking reaction was stopped by the addition of glycine to a final concentration of 0.125 M. Cells were washed in ice cold PBS and nuclei were isolated with cell lysis buffer (5 mM Pipes (pH 8.0), 85 mM Kcl, and 0.5% NP40). Nuclei were resuspended in nuclear lysis buffer (50 mM Tris (pH 8.0), 10 mM EDTA, and 1% SDS) and sonicated using a Branson 250 sonifier. Settings were optimized to yield a mean genomic DNA size of 0.2 to 0.5 kB. Chromatin was diluted 1∶3 in dilution buffer (0.01% SDS, 1% Triton-X100, 2 mM EDTA, 150 mM Nacl, and 20 mM Tris (pH 8.0), precleared with Staph A cells (BD) for 15 min at 4°C. Chromatin preparations obtained from 5×10^6^ cells were incubated in the presence of 1 µg of control goat IgG or anti-Gfi1 (N20; Santa Cruz Biotechnology) for 3 hours and precipitated using Staph-A cells. Upon washing of the immunoprecipitates, DNA was purified by phenol/chloroform extraction and proteinase K digestion. Input and immunoprecipitated DNA samples were analysed by semiquantitative PCR (35 cycles) with primers amplifying either the IL-7Rα intron 2 (forward primer 5′ GCCCACTGTAACAAACTTCCC, reverse primer 5′ GCCTATAAAGTTTGCAAGTCC) or IL-7Rα exon 8 specific primers (forward primer 5′ CTGGACTGCCAATTCATGAGGTG, reverse primer 5′ TCTCTGTAGTCAGGGGACCTAGAG) used as control. PCR products were separated by 1.7% agarose gel and visualised after staining with ethidium bromide.

### Statistical analysis

Data are presented as mean±SEM. Statistical significance was assessed using a 2-sided Student *t* test. *P* values >0.05 were considered to be non significant (NS) and *P* values <0.05 and >0.01 were represented as *. *P* values <0.01 and >0.001 were represented as ** and *P* values <0.001 were represented as ***.

## Supporting Information

Figure S1 Transcriptional activity of Gfi1 locus in developing B cells. A) Gfi1 expression in defined Hardy fractions. Pooled bone marrow cells from 5 mice were analysed for GFP expression in B220^+^CD43^+^BP1^−^ (Fraction A–B), B220^+^CD43^+^BP1^+^ (Fraction C–C'), B220^+^CD43^−^IgM^−^ (Fraction D), B220^+^CD43^−^IgM^+^ (Fraction E) and B220^high^CD43^−^IgM^high^ (Fraction F) cells. Shaded histograms represent GFP fluorescence in Gfi1^+/GFP^ cells, open histograms represent autofluorescence in Gfi1^+/+^ cells. The GMFI. of Gfi1^+/+^ (top) and Gfi1^+/GFP^ (bottom) cells is indicated. Data are representative of 3 independent experiments. B) Gfi-1 expression during in-vitro B cell development. LSK bone marrow cells from Gfi1^+/GFP^ mice were cultured in the presence of SCF and IL7. Cells were harvested at indicated time points and their GFP fluorescence was determined by flowcytometric analysis. Shown is the specific geometric mean fluorescence intensity index calculated as follows: GMFI_i_ = GMFI_(Gfi1_^+/GFP^)−GMFI_(Gfi1_^+/+^). Results represent the average values of duplicate samples. Data are representative of 2 independent experiments.
(0.18 MB PDF)

Figure S2 shRNA-mediated knockdown of Gfi1 in hematopoietic progenitor cells. HSC from Gfi1^+/+^ and Gfi1^−/−^ mice were sorted, cytokine-stimulated and transduced with lentiviral vectors (control backbone, sh-RNA1, or sh-RNA2, respectively). After 3 days in culture, cells were harvested and subjected to RT-PCR using Gfi1-specific and GAPDH-specific primer pairs.
(0.09 MB PDF)

Figure S3 IL7Rα expression levels in primary and in *in vitro* cultured hematopoietic progenitor cells. A & B. Hematopoietic progenitor cells from Gfi1^+/+^ and Gfi1^−/−^ mice were sorted and cultured in the presence of mIL3, mSCF, mIL6, mFlt3L and hTPO for 48 hours. Cells were stained with anti-IL7Rα antibodies and analyzed by flow cytometry. Note that IL7Rα expression was undetectable in non-stimulated HSCs
(0.27 MB PDF)

Figure S4 Proliferation assay of hematopoietic progenitor cells in response to cytokines (CFSE-assay). LSK cells from Gfi1^+/+^ and Gfi1^−/−^ mice were CSFE-labelled and incubated in the presence of cytokines for 72 hours. Histograms representing CFSE fluorescence and division history of Gfi1^+/+^ (top panel) and Gfi1^−/−^ (bottom panel) cells are shown. Data are representative of 2 independent experiments. Note that Gfi1^−/−^ cells cultured in the presence of a) IL-3+ SCF+ Flt3L+ IL-6+ TPO, b) SCF+ IL7 and c) SCF show similar proliferative responses.
(0.25 MB PDF)

Figure S5 Proliferation assay of HSC in response to cytokines (BrdU-assay). Sorted CD150^+^CD48^−^ cells from Gfi1^+/+^ and Gfi1^−/−^ mice were cultured in the presence of either SCF + IL7 or SCF and IL7 only for 60 hours. BrdU was added and the cells were cultured for additional 12 hours. Proliferation of cells was assessed by FACS upon anti-BrdU staining.
(0.23 MB PDF)

Figure S6 CFU assay determining the proliferative capacity of CD48^−^CD150^+^ HSC. CFU assay indicating decreased colony-forming-activity in Gfi1^−/−^ HSC. CD48^−^CD150^+^ cells were cultured on semisolid medium in the presence of indicated cytokines. 14 days later, the absolute numbers of colony forming units of Gfi1^+/+^ (white bars) and Gfi1^−/−^ (black bars) cells were enumerated and plotted.
(0.09 MB PDF)

Figure S7 Gating strategy and analysis of B cell specific transcription factor expression in Gfi1^+/+^ and Gfi1^−/−^ B cells. A) Total bone marrow cells of Gfi1^+/+^ and Gfi1^−/−^mice were stained with B220-specific antibodies and further analysed for expression of CD19 and IgM. Three fractions discriminated and designated as G1 (B220^+^CD19^−^IgM^−^), G2 (B220^+^CD19^+^IgM^−^) and G3 (B220^+^CD19^+^IgM^+^). Cells were sorted yielding purities of >95%. The plots were generated to indicate purity of cell populations for preparative purposes and do not reflect absolute numbers of B lineage cells in mice. The percentages of gated cell populations are as follows: In Gfi1^+/+^ G1 = 16%, G2 = 50%, G3 = 28%. In Gfi1^−/−^ G1 = 53%, G2 = 20% andG3 = 21%. B) Expression of B cell specific transcription factors in G1 (B220^+^CD19^−^IgM^−^), G2 (B220^+^CD19^+^IgM^−^) and G3 (B220^+^CD19^+^IgM^+^) B cell fractions. mRNA expression levels of E2A (top panel) EBF (middle panel) Pax5 (bottom panel) were determined by RT-PCR. Shown are the mean values of duplicate samples. Data are representative of 2 independent experiments.
(0.28 MB PDF)

Figure S8 IL7Rα expression in bone marrow B lineage cells. A) Nucleated bone marrow cells of Gfi1^+/+^ and Gfi1^−/−^ mice were stained with anti-B220, anti-CD19, anti-B220, and anti-IL7Rα specific antibodies and analysed by flowcytometry. B220^+^ cells were gated (G1; top panel) and further analysed for expression of CD19 and IgM, yielding three distinct fractions: G1 (B220^+^CD19^−^IgM^−^), G2 (B220^+^CD19^+^IgM^−^) and G3 (B220^+^CD19^+^IgM^+^). B) FACS plots indicating IL7Rα surface expression in B cells. Cells of G2 (top panel), G3 (middle panel) and G4 (bottom panel) gates of Gfi1^+/+^ and Gfi1^−/−^ mice were analysed for IL7Rα expression. The GMFI measuring IL7Rα expression is indicated in each plot.
(0.36 MB PDF)

Table S1 Average frequency of Hardy Fraction's in the BM of Gfi1^+/+^ and Gfi1^−/−^ mice.
(0.02 MB XLS)
